The article "Factors affecting weekday-to-weekend sleep differences among Korean adolescent students: Focus on extracurricular tutoring time" was published in 2021. Journal: PLoS One.

# Factors affecting weekday-to-weekend sleep differences among Korean adolescent students: Focus on extracurricular tutoring time

**DOI:** 10.1371/journal.pone.0259666

**Published:** 2021-11-18

**Authors:** Jin-Won Noh, Young Dae Kwon, Jooyoung Cheon, Jinseok Kim

**Affiliations:** 1 Department of Health Administration, Yonsei University, Wonju, Korea; 2 Department of Humanities and Social Medicine, College of Medicine and Catholic Institute for Healthcare Management, The Catholic University of Korea, Seoul, Korea; 3 Department of Nursing Science, Sungshin Women’s University, Seoul, Korea; 4 Department of Social Welfare, Seoul Women’s University, Seoul, Korea; IRCCS Istituto Delle Scienze Neurologiche di Bologna, ITALY

## Abstract

**Objectives:**

Discrepancy in weekday-weekend sleep induces negative effects on physical health, obesity, psychological disorders, and academic performance; this particularly affects adolescent students through extracurricular tutoring, including evening self-study, private tutoring, and home studies. The present research aimed to clarify sociodemographic and economic factors, including extracurricular tutoring time, associated with weekday-to-weekend sleep differences using longitudinal data.

**Study design:**

Data from the Korean Children and Youth Panel Survey (KCYPS) data were analyzed. Weekday-to-weekend sleep differences and extracurricular tutoring, as well as other covariates, were measured using adolescent’s self-report questionnaires. Multilevel regression and structural equation modeling (SEM) of repeated measures were used to test the hypothesized relationship between variables.

**Results:**

The time spent in weekly extracurricular tutoring was negatively associated with weekday-to-weekend sleep differences. However, increased tutoring time was positively associated with bedtime, and bedtime was in turn positively associated with differences in Korean adolescents’ weekday-to-weekend sleep patterns. The SEM analysis result showed a significant indirect effect of tutoring time on sleep differences via bedtime.

**Conclusions:**

Limiting weekly extracurricular tutoring time is important to early bedtime and reducing weekday-to-weekend sleep pattern differences. Policymakers should develop alternatives to private tutoring to improve the sleep duration and reduce weekday-to-weekend sleep differences among adolescents.

## Introduction

Many countries have confirmed that sleep problems among youth are a public health concern [1, 2]. Weekday-to-weekend sleep differences (ie, lack of consistency of bedtime and wake-up patterns between weekday and weekend) are characteristic of young populations. Many environmental and psychosocial factors contribute to weekday-to-weekend sleep differences [3]. One of these factors is increased eveningness. Increased eveningness is common among adolescents, and this leads to larger weekday and weekend sleep differences [4]. Indeed, change of sleep patterns occur in most adolescents [5]. The transition of the sleep-wake patterns due to pubertal development and higher level of school grade, and the eveningness were associated with insufficient sleep during school days. In adolescents, they were more likely to compensate sleep on weekends for sleep deficiency on weekdays. So, the shorter sleep duration on weekdays or weekends were related to weekday-to-weekend sleep differences.

There are few prior studies comparing weekday and weekend sleep patterns. Previous studies showed that low sleep quality due to the discrepancy in weekday-weekend sleep results in negative effects not only on physical health (including obesity) but also on mental health and academic performance [6]. Adolescents with differing sleep patterns between weekdays and weekends were more likely to engage in increased unhealthy behaviors such as smoking and alcohol consumption [7].

Discrepancy in sleep patterns can mainly be explained based on biological factors such as intrinsic circadian delay associated with the pubertal development and the mismatch between endogenous circadian timing and socio-environmental demands [2, 3, 8]. For example, the development of puberty which could induce delayed intrinsic circadian rhythm is likely to increase eveningness preferences, including a preference for a late bedtime and later wake-up time. Because adolescents must attend social activities like school on the weekdays, the increase of eveningness could be inconsistent with the social environment, so adolescents tend to sleep longer in weekends [4, 9–11]. Meanwhile, adolescents who engaged in extracurricular tutoring showed shorter sleep durations. Longer tutoring time was related with delayed bedtime [5]. Pressures from the sociocultural environment (including academics and social activities) thus induced weekday-weekend sleep differences [5, 6]. This sleep difference often results in social jetlag, which has been related to health and cognitive issues [2, 3, 8].

Previous studies have been limited in focus, with greater attention being paid to biological factors and social jetlag. More studies are therefore needed to consider other factors such as social demands. This study sought to clarify sociodemographic and economic factors, including extracurricular tutoring time, associated with weekday-to-weekend sleep differences among adolescent students using nation-wide longitudinal data. Using structural equation modeling (SEM) approach that presents combined model in factor analysis for theoretical association in structural model including potential or/and unobserved variables, this study tested the hypothesized relationship between extracurricular tutoring time and weekday-to-weekend sleep differences.

## Methods

### Data and participants

This study used data from the Korean Children and Youth Panel Survey (KCYPS). Based on a nationally representative sample of Korean children and youths from three different developmental stages, first (age 6) and fourth grade (age 9) elementary school students and first grade junior high school students (age 12), the KCYPS sought to better understand Korean youths’ growth and development. The KCYPS started in 2010 and continued data collection every year until 2016. The KCYPS implemented multi-stage stratified cluster sampling with schools as the primary sampling unit. The present study used data from the junior high school student panel (N = 2,351), including data from the first year of junior high school to the last year of high school and excluding the final year data when the respondents had graduated from high school. This study was approved by the Institutional Review Board of Seoul Women’s University (IRB-2018-46) with a waiver for informed consent because the data were obtained from a public data depository which is freely available online.

### Variables and measurements

Demographic and socio-economic characteristics of the adolescents including gender; family type (ie, living with both parents, living with single parent, or other); housing type (ie, house, apartment, and others); living area (ie, rural or urban); and socioeconomic status were included in this analysis. The socio-economic status of the adolescents was measured by parents’ job status and education level. Parental job status was measured by a question asking both parents whether they were working for pay. Parental education level was defined as whether they had earned a college degree. Parental job status and education level were asked for both parents and used as separate variables.

The weekday-to-weekend sleep difference variable was defined as the difference between the average sleep duration on weekdays and weekends in minutes. Sleep duration was calculated using the bedtime and wake-up times self-reported by the respondents. These times were measured by the following question: “What times do you usually fall asleep and get up?”, which were asked separately for weekdays and weekend days. Extracurricular tutoring time was measured by calculating the total amount of time per week the adolescents spent on tutoring activities in minutes.

### Statistical analysis

A series of descriptive statistics were provided to depict the overall characteristics of the sample. A multilevel model with repeated measures was used to account for the overestimation of standard errors in panel data [12]. A SEM was used to test the relationship among extracurricular tutoring time, bedtime, and weekday-to-weekend sleep difference for Korean adolescents. Stata 15 (StataCorp LP, College Station, Texas) was used to manage the data and analyze the models.

## Results

Table 1 summarizes the characteristics of the sample from Wave 1 during the first year of junior high school to Wave 6 at the third year of high school. There were about the same number of females and males in the sample. Under 10% of adolescents were living with a single parent (minimum: 7.9% [Wave 2], maximum: 9.5% [Wave 1]) and about 10% were living with grandparents or other family members (minimum: 7.1% [Wave 6], maximum: 12.3% [Wave 1]). About two thirds of mothers were working outside the home (minimum: 62.5% [Wave 1], maximum: 70.9% [Wave 5]) while over 90% of fathers were working outside the home (minimum: 90.4% [Wave 6], maximum: 98.4% [Wave 2]). About 60% of adolescents responded that both their parents were working (minimum: 58.8% [Wave 6], maximum: 68.1% [Wave 5]). The proportion of fathers with college or higher degree was around 45% (minimum: 40.7% [Wave 1], maximum: 46.2% [Wave 2]), while for mothers the proportion was around 30% (minimum: 26.0% [Wave 1], maximum: 32.8% [Wave 6]). Most adolescents were living in an apartment (minimum: 59.1% [Wave 1], maximum: 60.7% [Wave 3]), and about 20% were living in housing types other than a house or apartment (minimum: 14.6% [Wave 5], maximum: 20.3% [Wave 1]). Almost 90% of adolescents were living in urban areas (minimum: 84.2% [Wave 6], maximum: 85.8% [Wave 5]).

**Table 1:** Sample characteristics of Korean adolescent students.

	Wave 1		Wave 2		Wave 3		Wave 4		Wave 5		Wave 6	
	n	%	n	%	n	%	n	%	n	%	n	%
Gender: female	1,175	50.0	1,128	49.5	1,119	49.5	1,033	49.0	1,024	49.0	1,015	49.4
Family type: single parent	224	9.5	176	7.9	207	9.3	195	9.2	191	9.4	180	9.2
Family type: etc.	288	12.3	232	10.5	188	8.5	166	7.9	152	7.5	139	7.1
Mother working	1,376	62.5	1,401	67.3	1,422	68.3	1,350	68.3	1,346	70.9	1,269	65.1
Father working	2,101	96.5	2,018	98.4	1,999	97.4	1,909	97.4	1,820	97.5	1,761	90.4
Both parents working	1,211	59.1	1,266	64.9	1,262	65.0	1,220	65.8	1,203	68.1	1,140	58.8
Mother college graduate	571	26.0	676	32.6	676	32.4	642	32.5	619	32.6	602	32.8
Father college graduate	883	40.7	944	46.2	931	45.3	884	45.1	840	45.0	801	44.6
Housing type: apartment	1,385	59.1	1,327	59.8	1,349	60.7	1,249	59.2	1,226	60.4	1,188	60.6
Housing type: etc.	477	20.3	362	16.3	337	15.2	357	16.9	296	14.6	327	16.7
Living in urban area	2,014	85.7	1,895	85.4	1,929	85.4	1,801	85.4	1,743	85.8	1,652	84.2
	Mean	SD	Mean	SD	Mean	SD	Mean	SD	Mean	SD	Mean	SD
Sleep differences (minute)	96.8	102.4	103.7	101.1	106.2	96.9	133.2	103.4	132.6	99.5	116.2	100.2
Bedtime (hh:mm, minute)	23:7	56.1	23:21	56.1	23:40	59.2	0:17	62.3	0:34	63.1	0:31	67.0
Extracurricular tutoring (minute)	245.5	212.9	212.4	189.8	185.0	187.7	157.5	208.3	160.0	221.3	143.5	241.3

SD, standard deviation; The participants were at their first year of junior high school at Wave 1 and at third year of high school at Wave 6.

Throughout the study period, the adolescents reported from 96.8 minutes (SD = 102.4) at Wave 1 to 133.2 minutes (SD = 103.4) at Wave 4 of sleep difference between weekdays and weekends. The adolescents reported that their bedtime was around midnight (minimum: M [SD] = 23:07 [56.1] in Wave 1, maximum: M [SD] = 00:34 [63.1] in Wave 5). On average, the adolescents spent 2 to 4 hours per week on extracurricular tutoring time (minimum: M [SD] = 143.5 [241.3] minutes in Wave 6, maximum: M [SD] = 245.5 [212.9] minutes in Wave 1; see also Table 1).

Fig 1 illustrates the weekday-to-weekend sleep differences among Korean adolescent students over time during the study period. During the first three years of junior high school, the adolescents’ sleep differences tended to increase over time. In the year the adolescents made a transition from junior high to high school, a clear discontinuity was observed. After the sudden jump, the difference for the high school students presented an overall decrease over time (Fig 1). The amount of sleep difference between weekdays and weekends was further examined in association with a variety of adolescent characteristics. Results from a series of bivariate multilevel regression analyses are presented in Table 2. Female adolescents reported greater sleep difference than males (B [SE] = 34.69 [2.58], p<0.001). The adolescents living with family members other than their parents reported lower amount of sleep difference than youths living with both parents (B [SE] = -8.92 [3.76], p = 0.018). The adolescents living in an apartment (B [SE] = 9.63 [2.82], p = 0.001) reported larger sleep differences compared to house-dwellers, as did residents of urban areas (B [SE] = 7.53 [3.53], p = -0.033) compared to rural areas. The time spent in weekly extracurricular tutoring was negatively associated with weekday-to-weekend sleep differences (B [SE] = -1.38 [0.26], p<0.001). The same association was found for weekday tutoring time (B [SE] = -2.62 [0.45], p<0.001) and weekend tutoring time (B [SE] = -1.16 [0.45], p = 0.010; see Table 2).

**Fig 1:** Adolescents’ weekday-to-weekend sleep differences over time.

**Table 2:** Bivariate multilevel regression results showing relationship of weekday-to-weekend sleep differences and adolescent characteristics.

	B	SE (B)	95% CI
Gender (female)	34.69***	2.58	(29.64, 39.73)
Family type (single parent)	-1.24	4.00	(-9.08, 6.60)
Family type (etc.)	-8.92*	3.76	(-16.29, -1.56)
Father college graduate or higher	0.01	2.49	(-4.87, 4.89)
Mother college graduate or higher	-2.79	2.63	(-7.95, 2.37)
Mother working	0.19	2.38	(-4.49, 4.86)
Father working	-2.69	5.22	(-12.93, 7.55)
Both parents working	1.21	2.37	(-3.44, 5.85)
Living in urban area	7.53*	3.53	(0.61, 14.45)
Housing type (apartment)	9.63**	2.82	(4.10, 15.15)
Housing type (etc.)	4.39	3.30	(-2.07, 10.85)
Extracurricular tutoring time: total	-1.38***	0.26	(-1.90, -0.87)
Extracurricular tutoring time: weekday	-2.62***	0.45	(-3.50, -1.74)
Extracurricular tutoring time: weekend	-1.16*	0.45	(-2.05, -0.28)

*p<0.05,

**p<0.01,

***p<0.001.

To clarify the association between sleep difference and tutoring time for Korean adolescents, we tested a model with the bedtime of the adolescents in relation to sleep difference and extracurricular tutoring time. The results showed that increased tutoring time was positively associated with delayed bedtime (B [SE] = 0.58 [0.19], p = -0.002), and bedtime in turn was positively associated with weekday-to-weekend sleep differences (B [SE] = 0.48 [0.01], p<0.001). That is, adolescents spending more time on extracurricular tutoring would go to sleep later at night, and those who slept later would experience longer sleep differences between weekdays and weekends. This indirect effect of tutoring time on sleep difference via bedtime was significant (B [SE] = 0.28 [0.09], p = 0.002; see Table 3).

**Table 3:** Relationship between extracurricular tutoring time, bedtime, and weekday-to-weekend sleep difference.

Dependent Variable	Independent Variable	B	SE (B)	95% CI
Sleep difference	Bedtime	0.48***	0.01	(0.46, 0.51)
	Extracurricular tutoring time	-1.51***	0.25	(-2.00, -1.03)
Bedtime	Extracurricular tutoring time	0.58**	0.19	(0.21, 0.95)
Indirect effect	Extracurricular tutoring time—Bedtime—Sleep difference	0.28**	0.09	(0.10, 0.46)

SE, standard error; CI, confidence interval.

*p<0.05,

**p<0.01,

***p<0.001.

## Discussion

The present study investigated weekday-to-weekend sleep differences among adolescent students in South Korea. The sleep difference time was 1.6–2.3 hours, which was like the 1.8 hours found for Indian adolescents [13] and longer than the 1.2 hours found for US adolescents [14]. Sleep differences among junior high school students tended to increase over time, but a sudden jump appeared at the transition from junior high school to high school.

The large weekday-to-weekend sleep difference in high school students may be influenced by the increased duration of weekend catch-up sleep due to the unique program of the evening self-study at Korean high schools [15–17]. Most high school students generally start their classes at about 7:30–8:00 AM and participate in evening self-study sessions in which they could be monitored by teachers until 10 or 11 PM, while junior high school students stay at the school from about 8:00–8:30 AM to 4:00 PM. The evening self-study program could help students save study time, receive immediate help from their peers or the teachers, and get an advantage on their university entrance exams [15, 17]. However, such evening self-study programs tend to be compulsory, so students must stay at the school for up to 14 hours, which may lead to bad consequences such as a late bedtime, shorter sleep duration, and larger weekday-to-weekend sleep differences in high school students than among junior high school students [15–18].

The findings in this study also indicate that increased tutoring time was associated with a later bedtime, and a later bedtime was associated with an increase in weekday-to-weekend sleep differences. There could be several explanations for this. According to Korean Statistics from 2017 [19], 63.8% of junior high school students and 52.4% of high school students spent time in private tutoring or academic institutes for extracurricular studies. One study reported that the time for after-school classes, homework, and time on other learning activities were significant factors influencing decreased sleep duration both on school and non-school nights [20].

Interestingly, the increases in total extracurricular tutoring time were associated with a decrease in the weekday-to-weekend sleep difference even though the bedtime was still a significant factor associated with an increase in the weekday-to-weekend sleep difference. To understand better the nature of the relationship between sleep differences and extracurricular activities, it is necessary to carefully investigate the association of total extracurricular tutoring time, weekday extracurricular tutoring time, and weekend extracurricular tutoring time with weekday-to-weekend sleep differences.

The strength of the association between extracurricular tutoring time and sleep duration during weekend was stronger than the same during weekdays. If students spend time in extracurricular tutoring on the weekend, the weekday-to-weekend sleep difference decreases because the students lose the opportunity to make up for sleep deficiency. The weekday-to-weekend sleep difference increases if the students take extracurricular tutoring only on weekdays, which may result in late bedtimes on weekdays but not late on weekends. All in all, these results suggest that those students who spent weekend time in extracurricular tutoring were likely to curtail sleep duration both weekdays and weekend, which lead to decreased sleep differences. Their average sleep duration is expected to be less than those of students who only take extracurricular tutoring on weekdays. More tailored studies designed to investigate the association of sleep difference with extracurricular tutoring time and sleep duration stratified by weekdays and weekends are warranted.

The ordinance limiting the operating hours of “hagwons” (a for-profit private institute, academy, or cram school) to 10 PM in late 2010 may influence the transition from extracurricular tutoring on weekdays to weekend tutoring. One study found that since the ordinance was implemented, the average time spent on studying at hagwons between 10 PM to 12 AM decreased in 2014, but there was no significant difference in the change of sleep time and time spent in extracurricular tutoring [21]. The ordinance could not increase the sleep time and decrease the extracurricular tutoring time, but the pattern of going to hagwons at an earlier time on weekdays and even on weekends might have changed [21]. It seems that high school students who participated in the evening self-study sessions could not go to a private tutoring institute, so this might lead to the extracurricular tutoring time on weekend. Further investigations to compare several tutoring groups (eg, a group receiving extracurricular tutoring on weekdays, a group receiving extracurricular tutoring on weekend, and a group receiving extracurricular tutoring on both weekdays and the weekend) are required to determine the effect of private tutoring on weekday-to-weekend sleep differences.

In early 2010, the students’ human rights ordinance banning compulsory evening self-study at schools was enacted in some cities and provinces [16]. The ordinance decreased the spent in evening self-study. The ordinance did not lead to an increase in leisure time, however, but rather the hours for private tutoring and self-study outside schools increased. Students spent more than half of their leisure time on media use and games [16, 19]. Previous studies reported that bedtime use of technology was associated with reduced sleep quantity and quality and the development of health symptoms [22, 23]. Policymakers should encourage students to spend leisure time in a way conducive to their well-being and prevent a shift to additional private education hours.

There are several limitations to this study. First, sleep patterns were evaluated with self-reported data, which could lead to recall bias. Second, this study assessed the time spent sleeping, but did not evaluate sleep quality or other physical/psychological health problems that could affect sleep patterns. Last, time spent watching TV, gaming, using the Internet, and communicating using mobile devices on weekdays and weekends were not adjusted due to the lack of data. The present study was, however, meaningful in determining the effect of extracurricular tutoring time on weekday-to-weekend sleep differences among adolescent students in South Korea. Limiting extracurricular tutoring time on weekdays was important to encouraging early bedtimes, which reduces weekday-to-weekend sleep differences. However, the demand for extracurricular tutoring time may shift to increasing extracurricular tutoring time on weekends, which may influence total sleep quantity and quality. Policymakers should develop alternative options for private tutoring to satisfy students and their parents and reduce weekday-to-weekend sleep differences in terms of both quantity and quality of sleep.
